# The Effects of Phellodendron Decoction on Wound Healing of Anal Fistula after Anal Fistulotomy

**DOI:** 10.1155/2022/7363006

**Published:** 2022-07-22

**Authors:** Heng Deng, Jun Zhang, Xiancang Yuan

**Affiliations:** ^1^Department of Anorectal Surgery, Second Affiliated Hospital of Anhui University of Chinese Medicine, Hefei, China; ^2^Department of Basic Teaching and Research of Traditional Chinese Medicine, Anhui University of Traditional Chinese Medicine, Hefei, China; ^3^Department of Anorectal Surgery, Huainan City People's Hospital, Huainan, China

## Abstract

**Objective:**

To analyze the therapeutic effect of Compound Phellodendron decoction on wounds after anal fistulotomy.

**Methods:**

100 patients with anal fistula who underwent anal fistulotomy from April 2019 to April 2021 were included in the study group and control group according to the random number table method. 50 patients in the study group were treated with Compound Phellodendron decoction by fumigation and sitting bath, while warm water replaced Compound Phellodendron decoction in the control group. Perianal pain, wound edema, and exudation were scored on postoperative days 3 and 7, and wound healing time was recorded. Interleukin-2(IL-2), IL-5, IL-6, and IL-12 were measured via a double-antibody sandwich enzyme-linked immunosorbent assay. Hematoxylin-eosin (HE) staining and immunofluorescence were used to quantitatively analyze the capillary number and CD4+ and CD8+ lymphocytes in granulation tissue on postoperative days 7.

**Results:**

The scores of pain, edema, and exudation in 2 groups on postoperative day 7 were lower than those on the 3rd postoperative day. Compared with the control group, the pain, edema, and exudation scores in the study group were decreased, and the wound healing time was shortened; the expressions of IL-2 and IL-12 in the study group were significantly increased, while the expressions of IL-5 and IL-6 were decreased; the number of capillaries and CD4+ lymphocytes in the study group was increased, while the number of CD8+ lymphocytes was decreased.

**Conclusion:**

Compound Phellodendron decoction had efficacy in promoting wound healing, reducing complications, and changing lymphocyte aggregation and alleviating local inflammatory response.

## 1. Introduction

Anal fistula is one of the most common diseases in anorectal surgery. Delayed healing and other complications may occur in some patients, reducing the quality of life [1]. The healing status after anal fistula surgery is related to many factors, and the surgical method is only one aspect that affects the healing rate and recurrence rate after anal fistula surgery [2, 3]. The nutritional status of patients and the local microenvironment of wounds are also important factors affecting healing, such as systemic hyperglycemia in diabetes patients [4] and local inflammation of Crohn's anal fistula. The immuno-inflammatory response is a prerequisite for wound healing and tissue regeneration [5]. Systemic and topical immune regulation could improve the health status of patients and the healing environment of local wounds [6]. Lymphocyte count is an effective predictor of body nutrition, immune status, and inflammatory response [7]. Patients with a reduced systemic lymphocyte count often suffer from immune disorders whose healing ability of incisions or wounds is decreased [8]. However, lymphocyte aggregation and the change of subtype ratio in the local wound are also important manifestations of the inflammatory response, which can often delay healing [9]. Changes in systemic lymphocytes and their subsets have important significance in predicting systemic infection and the risk of related death [10]. However, the association between local lymphocyte count in the wound and the healing time of the wound after anal fistulotomy remains unclear.

Traditional Chinese medicine has a long history in the treatment of anal fistula, which can not only relieve postoperative pain but also significantly shorten the course of the disease [11]. Compound Phellodendron decoction has the functions of clearing, reducing swelling, and relieving pain [12], astringent, and hemostasis. It mainly improves local blood circulation around the anus, reduces edema, exudation, and other adverse factors of wound healing, and alleviates spasms and pain in the sphincter of patients through local heat fumigation and washing [13]. The aims of this study are to observe the influence of lymphocyte subsets in granulation tissue and to elucidate the curative effect of Compound Phellodendron decoction on wound healing.

## 2. Material and Methods

### 2.1. Clinical Data

The experiment was approved by the Ethics Committee of the Second Affiliated Hospital of Anhui University of Chinese Medicine (committee approval number: 2022-zj-19) and informed consent was obtained. The clinical data of 100 patients with anal fistula who underwent surgical treatment in the Anorectal Surgery Department of the Second Affiliated Hospital of Anhui University of Traditional Chinese Medicine from April 2019 to April 2021 were collected (Figure 1). The inclusion criteria for anal fistula patients were: ① definite anal fistula diagnosis; ② complete clinical data. Exclusion criteria: ① the diagnosis of anal fistula is not clear; ② combined with anorectal tumor; ③ anal fistula complicated with acute infection; ④ patients with tuberculosis and Crohn's disease; ⑤ patients with hematologic diseases; ⑥ patients allergic to traditional Chinese medicine. A total of 100 cases were included, including 77 males and 23 females, aged from 19 to 71 years old, with an average age of 40.23 ± 12.61 years old. There were 24 cases of high anal fistula and 76 cases of low anal fistula (Table 1).

### 2.2. Test Grouping

The general situation of patients and anal fistula type were collected, and health education and routine examinations were carried out. According to the numerical table method, patients were randomly divided into a control group and a study group, with 50 cases in each group. Control group: 37 males and 13 females, aged 19–66 years, with an average age of (39.53 ± 12.96) years. Study group: male 40 cases, female 10 cases; the age ranged from 22 to 71 years, with an average age of (41.25 ± 10.53) years. There were no significant differences in sex, age, anal fistula type, and other general conditions between the two groups (sex: *χ*2 = 2.181, *P*=0.235; age: *T* = 0.802, *P*=0.396).

### 2.3. The Preparation of Compound Phellodendron Decoction

Dried herbs with a total weight of 100 g (including *Phellodendri Chinensis Cortex* 30 g, *Sophorae flavescentis Radix* 25 g, *Salviae miltiorrhizae* 15 g, *Bletillae rhizoma* 10 g, and *Angelicae dahuricae Radix* 20 g) were soaked in 1 liter of cold water for 20 minutes and decocted in an automatic high-pressure airtight decocting machine (JMC-25 L, Jimi Factory, Zhengzhou, China) for 30 minutes. 400 ml of Compound Phellodendron decoction was obtained, sealed, and divided into 200 ml sterile plastic bags for use. The crude drug concentration is 0.25 g/ml.

General microbial check of decoction: From 1 bag of decoction sample of Phellodendri packed, shaken well, 10 ml sample solution was absorbed into a sterilized, tightly capped container containing 100 ml protein glue buffer (Chuangsai Technology Co., LTD, Shanghai, China) of pH 7.0 sodium chloride. The total number of aerobic bacteria, molds, and yeasts was counted by the medium dilution method (0.2 ml/dish).

### 2.4. Treatment

All the patients received conventional surgical treatment according to the type of anal fistula, followed by fumigation and sitz bath treatment via fumigating and sitting bath apparatus (model TM50-C, from Tianma Medical Instrument Factory, Xuzhou, China) on the second day postoperatively, once a day for 12 minutes (Figure 2). During dressing change, pay attention to the hyperplasia of granulation on the wound surface. The excessive growth of granulation tissue should be cut off to guard against pseudo healing. Control group: 2 liters of warm water cooled naturally to 40°C is used for fumigation and sitz bath treatments. Study group: 200 ml Compound Phellodendron decoction was added to 1.8 L of warm water at 40°C for the fumigating and sitz bath.

### 2.5. The Curative Effect and Index Were Observed

Wound edema, local pain, and exudation were measured on day 3 and 7 after surgery. At the same time, granulation wound edema and exudation were scored with 0∼3 points. (0: no edema or no exudation; 1: the edematous or exudate area is less than 1/4 of the wound area; 2 : 1/4–1/2, 3: the edematous or exudate area is greater than 1/2). The pain was assessed by Visual analogue scale (VAS), with a score of 0–10, 0 indicating no pain. The complete healing time of the anal fistula wound was recorded. Cure standard according to “Traditional Chinese Medicine disease diagnosis and Curative effect standard.” The absence of tenderness and scarring of surgical wounds on the skin of all fistula areas, and the absence of any drainage of pus from conduits or anus, are considered criteria for complete clinical healing of anal fistulas [14].

### 2.6. Hematoxylin-Eosin Staining (HE Staining)

The granulation specimens were cut at dressing change on the 3rd and 7th day after surgery and fixed with 10% formalin fixative. After dehydration, the granulation specimens were embedded in a paraffin embedding machine (Yaguang YB-7B, Xiaogan, China). The thin slices with a thickness of 5–8 microns were cut by a slicing machine (Leica RM2135, Heidelberg, Germany), pasted on slides, and dried in a 45°C thermostat (Fuma GHX-9270B-1, Shanghai, China). They were dyed in hematoxylin aqueous solution and eosin staining solution. The microscope (Nikon 80i, Tokyo, Japan) randomly selected 3 fields in each section to count capillaries.

### 2.7. Double Antibody Sandwich Enzyme Linked Immunosorbent Assay (ELISA)

The enzyme-plate analyzer (Model RT-6000, Redu, Shenzhen, China) was used to quantitatively detect the expressions of interleukin-2, IL-5, IL-6, and IL-12 in granulation specimens on the 3rd and 7th day after surgery. ELISA kits (Invitrogen, New York, USA) for human IL-2, IL-5, IL-6, and IL-12 were purchased from Hefei Linmei Biological Co., LTD.

### 2.8. Immunofluorescence

Immunofluorescence was used to qualitatively and quantitatively detect the expression of CD4+ and CD8+ in the granulation samples taken during dressing change on the 7th postoperative day. Three field counts were randomly selected for each section. The detection procedure was carried out according to the instructions of the PE kit (Becton and Dickinson Company, New York, USA), which was purchased from Hefei Linmei Biological Co., LTD.

### 2.9. Statistical Methods

Shapiro–Wilk test was employed to evaluated whether the data were normally distributed. Normal distribution measurement data were expressed as mean ± standard deviation (Mean ± SD). Descriptive statistics were used to analyze data on population characteristics, and the occurrence of complications. A paired sample *T*-test was utilized to compare the data of the same patient on postoperative days 3 and 7. A Levene test is performed to determine the homogeneity of variance. One-way ANOVA was performed to explore if mean absolute difference in the control group differed to the study group. Data were analyzed using R3.6.1 and Empower STATS software, and *P* < 0.05 was statistically significant.

## 3. Result

### 3.1. General Characteristics

There was no statistical significance in sex, age, anal fistula type, operation time, and other general characteristics between the study group and the control group (*P* > 0.05).

Comparison of postoperative complications (wound edema, pain, and exudation) between the two groups.

On the 3rd and 7th days after the operation, the scores of complications such as edema of the wound edge, anal pain, and wound exudation in the study group were lower than those in the control group. As shown in Figure 3, intuitively, the wound exudation in the study group was significantly lower than that in the control group. The complication scores of wound edema, anal pain, wound exudation, and other complications in both groups on the 7th day after surgery were lower than those on the 3rd day after surgery, with statistical significance (*P* < 0.05), as shown in Table 2.

### 3.2. Comparison of Wound Healing Time and Lymphocyte Subtype Number

The total healing time of anal fistula wounds in the study group (40.23 ± 9.61) was significantly lower than that in the control group (45.84 ± 13.29) (*P* < 0.05). The comparison in Figure 4 shows that the postoperative wounds in the study group healed completely earlier. But there was no statistical difference in the total healing rate between the groups. CD4+ and CD8+ subtypes of lymphocytes were positively expressed in the granulation tissues of patients in both groups. Compared with the control group, the number of CD4+ lymphocytes in the study group was significantly increased, while the number of CD8+ lymphocytes was significantly decreased (*P* < 0.05) (Table 3, Figure 5).

### 3.3. Expression of IL-2, IL-5, IL-6, and IL-12 in Granulation Tissue

The levels of IL-2 and IL-12 in granulation tissue of both groups on the 7th day were higher than those on the 3rd day. The levels of IL-5 and IL-6 in the granulation tissue of the study group on the 7th postoperative day were lower than those on the 3rd postoperative day. In the control group, IL-6 and IL-6 in granulation tissue on the 7th day after operation were higher than those on the 3rd postoperative day. Compared with the control group, the expressions of IL-2 and IL-12 in granulation tissue of the study group were significantly increased on the 7th postoperative day, while the expressions of IL-5 and IL-6 were decreased (*P* < 0.05) (Table 4).

### 3.4. The Number of Capillaries in Granulation Tissue Was Compared between the Two Groups

The number of capillaries in granulation tissue in both groups increased on the 7th day after the operation compared with the 3rd day (*P* < 0.05). Compared with the control group, the number of granulation tissue capillaries in the study group increased significantly on the 3rd and 7th postoperative days (*P* < 0.05) (Figures 6 and 7).

### 3.5. Discuss

The results of this study showed that the fumigation and washing of Compound Phellodendron decoction in the treatment of anal fistula could effectively reduce postoperative wound pain, exudation, and edema and other complications, and shorten the postoperative wound healing time of patients. Through data collection and immunofluorescence experiments, it was found that the number of CD4+ lymphocytes in the wound granulation tissue of anal fistula patients was negatively correlated with the healing time, while the increased number of CD8+ lymphocytes delayed the healing time. Fumigating-washing local wounds of anal fistula with Compound Phellodendron decoction is beneficial to reverse this trend, to change the aggregation of lymphocyte subtypes in granulation tissue, to improve the immune environment, and to promote the growth of capillaries in granulation tissue.

Lymphocyte subsets as markers to predict the prognosis and outcome of diseases have become the research direction of many scholars. Nunez et al. [15] found that in patients with acute coronary syndrome older than 65 years old, reduced lymphocyte count is a marker of inflammatory response and immunosuppression, which can be used to predict the weakened state of patients, and reduced lymphocyte count is independently associated with death, disease recurrence, and readmission. However, the significance of lymphocyte subsets in local tissues differs from that in serum and often reflects the severity of inflammation. Peng et al. [16] observed the infiltration of lymphocyte subsets into local wounds of burn patients and found that skin injury was closely related to the activation degree of local lymphocyte subsets. IL-2 and IL-12, which are mainly involved in cellular immunity, are secreted by CD4+ T lymphocytes. Il-5 and IL-6 cytokines, which are mainly involved in humoral immune responses, are secreted by CD8+T lymphocytes. [17] The expression of these inflammatory cytokines in serum often indicates the degree of the systemic inflammatory response, and the higher the expression level, the more severe the inflammatory response and the worse the prognosis. The higher the expression level of IL-2 and other inflammatory factors in the serum of patients with more severe craniocerebral injury [18]. Serum IL-6 and IL-2 were associated with adverse clinical features and worse outcomes in diffuse large B-cell lymphoma. However, these inflammatory cytokines (IL-2, IL-12, IL-5, and IL-6) have different effects on local wound healing [19, 20]. IL-2 and IL-12 produced by local wound tissue may play an important role in promoting their healing. IL-2 expression in granulation tissue of chronic ulcer wounds was positively proportional to the number of new capillaries, which significantly promoted ulcer healing [21]. IL-2 in local wounds can promote endothelial cell growth and angiogenesis in the mucosal wound [22]. Il-12 produced by local tissues can protect damaged skin [23]. The decrease of IL-5 and IL-6 in the granulation tissue of patients in the study group can reduce the local inflammatory response and inflammatory exudation related to humoral immunity. The mechanism may be to increase the local accumulation of CD4+ lymphocytes and to decrease the number of CD8+ lymphocytes in the wound, so as to increase the expression of IL-2 and IL-12 in the wound and promote the capillary hyperplasia of granulation tissue.

There is a long history of treating anal fistula with traditional Chinese medicine decoctions fumigating and sitting baths. This study was to observe the therapeutic effect of Compound Phellodendron decoction on wound healing after anal fistulotomy. Phellodendron, as the king of this prescription, was used for promoting wound healing. Phellodendron is the dried bark of Phellodendron chinense Schneid, a genus of Berberis in the Rue family. Liu et al. [12] evaluated Phellodendron in the treatment of diabetic foot ulcers and proved that it has the effect of improving VEGF, which can promote granulation growth. Not only can the drug itself reduce wound exudation but it can also promote other drugs to be absorbed through the skin. Wu et al. [24] used Phellodendron to treat burn wounds and proved that it could prevent infection during treatment. Phellodendron can activate the TGF-*β* signaling pathway and increase the expression of collagen during wound healing [25]. In the same way, as the minister, assistant, and envoy in the prescription, *Sophora flavescens*, *Salvia miltiorrhiza*, *Bletilla striata*, and *Angelica dahurica* have important effects on wound healing. Fan et al. [26] used *Sophora flavescens* and *Bletilla striata* to heal wounds of ulcerative colitis wounds as effectively as mesalazine. An anal fistula wound is a polluted wound, affected by defecation, whose surface has a variety of bacteria. Based on previous studies, Compound Phellodendron decoction is very suitable for promoting anal fistula wound healing. But the mechanism is unclear. In our study, Compound Phellodendron decoction was used to treat three types of surgical incisions that might be contaminated with feces. Instead of focusing on its bactericidal effect, the study elucidated its possible mechanism by regulating the proportion of local immune cells.

However, the molecular mechanism affecting the increase and decrease of lymphocyte subtypes remains to be further studied. The length of fumigation-washing time is only determined according to experience in the experiment, which may be a variable that changes the experimental results. Due to the large number of active ingredients in compound potion, the pharmacological properties of specific interventions have not been evaluated. Further experiments are needed to determine the defects mentioned above.

## 4. Conclusion

We verified the clinical therapeutic effect of Compound Phellodendron decoction on wound surface through fumigation-washing incision after anal fistulotomy. The mechanism of Compound Phellodendron decoction reducing postoperative wound pain, exudation and edema and shortening wound healing time may be to change the proportion of CD4+ and CD8+ lymphocytes in wound and promote capillary hyperplasia of granulation tissue.

## Figures and Tables

**Figure 1:** The diagram of participant flow describing the screening, randomization, allocation, and completion.

**Figure 2:** The fumigation and sitting bath treatment with Compound Phellodendron decoction. (a) The temperature can be adjusted by the fumigating and sitting bath apparatus. (b) The Compound Phellodendron decoction was continuously heated and exposed to the anal fistula wound.

**Figure 3:** The wound photos of the two patients on the 3rd and 7th day after surgery. (a) In the study group, the wound surface was moist on the third day after surgery, but the skin exudation around the wound surface had dried up. (b) In the study group, the degree of wound wetness on the 7th postoperative day was less than that on the 3rd postoperative day. (c) On the third day after surgery, the wound surface of the control group was oozing, accompanied by a large area of surrounding skin wet. (d) Fluid that can flow is still visible on the surface of the wound, although there is no obvious fluid in the skin surrounding the wound.

**Figure 4:** The wound photos of the two patients on the 42th day after surgery. (a) Surgical wounds in the study group were completely healed on the 42nd postoperative day. (b) Wounds in the control group tended to heal on the 42nd postoperative day.

**Figure 5:** The comparison of immunofluorescence expression images of CD4+ and CD8+ lymphocytes in wound granulation tissue between the study group with the control group. Compared with the control group (c) and (d), the number of CD4+ lymphocytes in the study group (a) was significantly increased, while the number of CD8+ lymphocytes (b) was significantly decreased.

**Figure 6:** The comparison of the number of capillaries in wound granulation tissue between the two groups. Compared with the control group (c) and (d), the number of capillaries in the study group (a) and (b) was significantly increased. The number of capillaries on day 7 (b) and (d) was larger than that on day 3 (a) and (c) in both groups.

**Figure 7:** The number comparison chart of capillaries in wound granulation tissue between the two groups. Compared with the control group, the capillary count in the granulation tissue stained by HE staining in the study group was significantly higher (^*∗*^: *P* < 0.05).

**Table 1:** Comparison of general data between the study group and control group (mean ± SD).

Item	Study group (*n* = 50)	Control group (*n* = 50)
Sex (M/F)	40/10a	37/13
Age	41.25 ± 10.53	39.53 ± 12.96
Length of fistula (cm)	3.1 ± 0.2	3.0 ± 0.3
Anal fistula type (complex/simple)	12/38	9/41
Operation time (Mins)	27.5 ± 3.3	25.2 ± 4.9

**Table 2:** Comparison of complications between the study group and control group (mean ± SD).

Postoperative complications	Study group (*n* = 50)		Control group (*n* = 50)	
	3rd	7th	3rd	7th
Edema	2.02 ± 0.33^#^	1.56 ± 0.27^*∗*^^#^	2.30 ± 0.21	1.86 ± 0.29^*∗*^
Pain	6.36 ± 1.04^#^	3.98 ± 0.87^*∗*^^#^	7.82 ± 1.73	5.09 ± 1.07^*∗*^
Effusion	2.26 ± 0.41^#^	1.35 ± 0.29^*∗*^^#^	2.82 ± 0.47	1.77 ± 0.36^*∗*^

**Table 3:** Comparison of wound healing and lymphocyte subtypes between the two groups.

Groups	Healing		Lymphocyte subtype	
	Healing time (day)	Number of recovered patients (cases)	CD4+ (/3HP)	CD8+ (/3HP)
Study group (*n* = 50)	40.23 ± 9.61	50	173 ± 36.5	89 ± 27.4
Control group (*n* = 50)	45.84 ± 13.29	49	125 ± 33.1	129 ± 20.2
*P*	0.0316	0.6778	<0.0001	0.0013

**Table 4:** Expressions of IL-2, IL-5, IL-6, and IL-12 in postoperative granulation tissue (Unit: ng·g^−1^).

Groups	Postoperative day 3				Postoperative day 7			
	IL-2	IL-12	IL-5	IL-6	IL-2	IL-12	IL-5	IL-6
Study group (*n* = 50)	50.36 ± 6.35	37.82 ± 8.81	98.61 ± 9.97	77.49 ± 7.91^#^	67.83 ± 3.15^*∗*^^#^	53.04 ± 5.72^*∗*^^#^	81.38 ± 8.94^*∗*^^#^	64.19 ± 6.56^*∗*^^#^
Control group (*n* = 50)	50.04 ± 7.02	35.08 ± 8.02	100.71 ± 8.98	94.35 ± 9.06	51.35 ± 5.36	44.78 ± 6.25^*∗*^	102.64 ± 10.42	97.08 ± 9.85

## Data Availability

The data that support the findings of this study are available from the corresponding author upon reasonable request.
